# Is There a Role for Probiotics in Liver Disease?

**DOI:** 10.1155/2014/874768

**Published:** 2014-11-11

**Authors:** Robert S. Lo, Andrew S. Austin, Jan G. Freeman

**Affiliations:** Liver Unit, Royal Derby Hospital, Derby DE22 3NE, UK

## Abstract

Intestinal microbiota plays an important role in health and disease. Alteration in its healthy homeostasis may result in the development of numerous liver disorders including complications of liver cirrhosis. On the other hand, restoration and modulation of intestinal flora through the use of probiotics is potentially an emerging therapeutic strategy. There is mounting evidence that probiotics are effective in the treatment of covert and overt hepatic encephalopathy, as well as in the prevention of recurrence of encephalopathy. The beneficial effect of probiotics also extends to liver function in cirrhosis, nonalcoholic fatty liver disease, and alcoholic liver disease. On the other hand, data associating probiotics and portal hypertension is scanty and conflicting. Probiotic therapy has also not been shown to prevent primary or secondary spontaneous bacterial peritonitis. Larger clinical studies are required before probiotics can be recommended as a treatment modality in liver diseases.

## 1. Introduction

Probiotics are defined by the World Health Organisation as live microorganisms that confer a health benefit on the host when administered in adequate amounts [1]. The concept of probiotics is not a novel entity. More than a century ago, Nobel Prize winner Eli Metchnikoff suggested that the long life of Bulgarian peasants was the result of their consumption of fermented milk products [2]. He went on to introduce in his diet sour milk fermented with the bacteria he called “Bulgarian Bacillus” and found his health benefited [3]. In actual fact, the practice of using probiotics in daily lives for health enrichment has been around for millenniums. Even in the ancient Greek and Roman empires, the use of cheese and fermented products was highly recommended [4]. Although the term “probiotic” was credited to Lilly and Stillwell [5] who in 1965 described probiotics as microorganisms that have effects on other microorganisms, the modern terminology and definition of probiotics was coined by Parker [6] who in 1974 defined probiotics as organisms and substances that have a beneficial effect on the host animal by contributing to its intestinal microbial balance. Consumption of modern era probiotics has been prevalent for decades even before the proper terminology was well established. As early as 1930, Shirota in Japan started to culture lactic acid bacteria (*Lactobacillus casei* strain Shirota) which he subsequently introduced into the market as Yakult in 1935 [7]. Today Yakult is marketed in 33 countries and 30 million bottles are consumed on a daily basis.

This review of probiotic use and liver diseases focuses on the following aspects: prevention of infection, hepatic encephalopathy, liver function in cirrhosis, nonalcoholic fatty liver disease, alcoholic liver disease, and portal hypertension.

## 2. Intestinal Microflora

There is a strong relationship between liver and the gut—the so-called Liver-Gut axis. The gut supplies blood to the portal system and intestinal blood content activates liver functions. On the other hand, the liver secretes bile and influences intestinal function [8].

Intestinal microflora forms a complex ecological system. It contains a large amount of microbes that weigh more than 1 kg. This quantity exceeds the number of cells in the human body 10-fold. The microbial community of the intestine consists of more than 500 species, most of which have not been cultivated, and many have yet to be identified. The intestinal microflora contains both bacteria that are fixed in the intestine (autochthonous, resident) and bacteria that only pass through the intestine (transient allochthonous) [9]. Most of the bacteria in the intestine form an anaerobic bioreactor that helps to digest difficult polysaccharides and synthesizes micronutrients including vitamins and short-chain fatty acids. The fermentation products of these bacteria can provide up to 10% of the daily energy needed by an individual [10].

The intestinal microflora has a variety of important physiological functions. It produces vitamins, degrades bile acids, digests nutrients, and forms important barrier against pathogens by producing local and general immunity [11].

In patients with liver cirrhosis, abnormal colonisation of the small intestine with colonic bacteria is well established. At least 50% have intestinal bacterial overgrowth. This is in comparison with healthy individuals who have only small amount of these bacteria in the small intestine. The main causes are thought to be hypochlorhydria, a decrease in IgA secretion, a decrease in intestinal motility, and malnutrition. In the clinical setting, increasing small intestinal motility pharmacologically with Cisapride has been shown to reduce bacterial overgrowth in patients with cirrhosis [12]. With such a close relationship between the liver and the gut flora, it is not surprising that many have postulated a role for gut barrier in the pathogenesis of liver diseases and its complications.

## 3. Bacterial Translocation

Bacterial translocation is defined as the migration of bacteria from the intestinal lumen to mesenteric lymph nodes of other extraintestinal sites [13]. The most effective bacteria to translocate to the mesenteric lymph nodes are Gram-negative members of the Enterobacteriaceae family such as* Escherichia coli* and* Klebsiella* spp,* enterococci*, and other* streptococci* species [14]. In an animal study, the prevalence of bacterial translocation to mesenteric lymph nodes is around 40% in cirrhotic rats with ascites [15] and around 80% in such animals with spontaneous bacterial peritonitis [16]. Available evidence has suggested that bacteria isolated from the mesenteric lymph nodes are genetically identical to strains causing spontaneous bacterial peritonitis (SBP) in the same animal [17]. In patients undergoing liver transplantation or liver resection, positive mesenteric lymph node culture for enteric bacteria was found in nearly 31% of Child-Pugh class C cirrhotics, which was 5 times higher than in Child Pugh Class A or B [18]. In cirrhotic patients undergoing partial hepatectomy, almost 20% were found to have positive mesenteric lymph node culture, and most of the postoperative infections were due to the same bacteria [19].

Bacterial DNA is found in approximately one-third of cirrhotic patients with portal hypertension and culture negative ascites, with* Escherichia coli* being the most frequently identified bacterial species [20]. The presence of bacterial DNA is associated with increased local levels of proinflammatory cytokines, which may be clinically significant [21]. Endotoxaemia is also postulated to increase portal pressure and impair haemostasis [22], as well as helping in the induction of variceal bleeding [23].

The pathogenesis of bacterial translocation in cirrhosis is complex. Apart from intestinal bacterial overgrowth, cirrhotics also exhibit changes in intestinal mucosa and intestinal immunity. Nitric oxide contributes to the morphological changes of the intestinal wall as it dilates tight junctions in cultured intestinal epithelial cells [24]. This represents the breaching of the first line of mucosal defence against paracellular absorption and hence the increased potential for bacterial translocation. Dilatation of the intercellular space below tight junctions, which is the second line of defence against paracellular absorption, also occurs in cirrhotics [25]. Thick-walled, dilated capillaries together with oedema of the lamina propria, fibromuscular proliferation, a reduced villous/crypt ratio, and thickened muscularis mucosa in the small bowel are found in cirrhotics [26] and have been proposed to play a role in bacterial translocation [27]. In addition intestinal immunity is also compromised. An animal study demonstrated an increased number of intraepithelial lymphocytes with markedly impaired proliferative activity and capacity for production of interferon-*γ*, correlating with increased bacterial translocation [28]. To summarise, the main mechanisms leading to bacterial translocation are bacterial overgrowth, a deficit in the local immune response of the mucous membrane, a decrease in phagocytic activity of macrophages as well as neutrophils, and an increase in the permeability of the intestinal barrier [29].

## 4. Probiotics: Mechanisms of Benefit

Mechanisms for the benefits of probiotics are not completely understood. However, four general benefits have been described [30]:

1. suppression of growth, epithelial binding, or invasion by pathogenic bacteria [31],
2. improvement of intestinal barrier function [32],
3. modulation of the immune system; these include the inducement of protective cytokines such as IL-10 [33] and TGF-beta and suppression of proinflammatory cytokines such as TNF [34]; suppression of T-Helper 1 cells migration has also been described [35],
4. modulation of intestinal pain perception by inducing expression of microopioid and cannabinoid receptors [36].

## 5. Prevention of Infection

Spontaneous bacterial infections such as SBP and bacteraemia are common in hospitalised cirrhotic patients. They also correlate with the severity of liver cirrhosis. These infections are associated with significant morbidity and mortality. For example, the prevalence of SBP in cirrhotic hospitalised patients with ascites is as high as 30% [37], and despite aggressive therapy, 1 in 5 patients still die from SBP [38].

The causal link between bacterial translocation and SBP has been well demonstrated [17]. Probiotic usage in this setting is attractive because of its ability to modulate gut flora, favouring protective anaerobic organisms, and also because of its effects in promoting gut barrier function [39]. Probiotic supplementation increases resistance to enteric infection in IL-10 deficient mice [17]. In clinical studies, probiotics have demonstrated efficacy in reducing endotoxaemia in cirrhotics [40], which is an indicator of the bacterial translocation, by reducing the viable counts of potentially pathogenic Gram-positive and Gram-negative gut flora in patients with cirrhosis [41]. Probiotics also reduce infections after orthotopic liver transplantation [42].

Current literature, albeit scanty, does not support the notion that probiotics prevent the occurrence of SBP. Using cirrhotic rats with ascites, probiotics failed to prevent bacterial translocation and ascitic fluid infection in spite of successful intestinal colonisation [43]. A recent clinical study showed that the addition of probiotics to norfloxacin did not improve its efficacy in preventing primary or secondary SBP or in reducing the mortality in cirrhotic patients with ascites [44].

## 6. Hepatic Encephalopathy

Gut microflora-derived ammonia has been widely recognised as the major contributor to the pathogenesis of hepatic encephalopathy. Modulating the intestinal flora pharmacologically remains the mainstay of treatments currently. This includes lactulose and nonabsorbable antibiotics such as neomycin and rifaximin.

As early as 1965, the idea of populating the colonic lumen with non-urease-producing bacteria as a treatment for hepatic encephalopathy was first put to test. An uncontrolled study suggested that high oral doses of* Lactobacillus acidophilus* might have a beneficial effect in patients with decompensated cirrhosis and hepatic encephalopathy [45]. Subsequently* Lactobacillus acidophilus* was shown to offer clinical improvement in encephalopathic patients refractory to neomycin alone [46]. Probiotics have been shown to reduce serum ammonia levels and result in improvement in various neurocognitive tests, as well as improvements in mental status [47].

A combination of prebiotics and probiotics (symbiotic approach) improved minimal hepatic encephalopathy, as well as reducing Gram-negative organisms in decompensated cirrhotics. A secondary end point for patients receiving symbiotic therapy was an improvement in overall liver function, as measured by the Child-Pugh score [48]. Similarly* Bifidobacterium longum* use in cirrhotic patients improves both minimal [49] and overt [50] hepatic encephalopathy. The use of probiotics in common clinical practice, however, requires further studies. A recent Cochrane review concluded that current available trials suffered from a high risk of bias and play of chance [51]. Although probiotics did appear to reduce plasma ammonia concentration, probiotics could not be concluded to be efficacious in altering clinically relevant outcomes.

The efficacy of probiotics in compensated cirrhotic patients with minimal hepatic encephalopathy has been studied. Treatment with probiotics preparation containing* Lactobacillus acidophilus*,* Lactobacillus rhamnosus*,* Bifidobacterium longum*, and* Saccharomyces boulardii* failed to produce any significant improvement in the various parameters assessed in patients with minimal hepatic encephalopathy, when compared with placebo [52]. Contrary to these studies, another study produced contrasting results demonstrating that three months of probiotics administration with VSL#3, which is a cocktail of probiotics, was effective in preventing HE in patients with cirrhosis as it significantly reduced levels of arterial ammonia, SIBO, and orocaecal transit time together with increased psychometric hepatic encephalopathy scores, compared with baseline [53].

The role of probiotics in secondary prophylaxis of HE has also been examined. Compared to placebo, treatment with probiotics conferred the same significant beneficial effect as lactulose in reducing HE recurrence over a 12-month follow-up [54].

## 7. Liver Function in Cirrhosis

Available studies suggest that probiotic therapy may improve liver function parameters in cirrhotic patients. In the study of synbiotic therapy described earlier [48], improvement of Child-Pugh class was recorded in nearly half the patients randomised to taking synbiotic therapy. The authors speculated that the improvement was secondary to the reduction in serum endotoxin levels. Using* Escherichia coli* Nissle, similar, but statistically less robust, results were achieved [40]. Patients treated with this probiotic for 42 days demonstrated a trend towards lower endotoxin levels and improvement in Child-Pugh score, although they were not statistically significant. Improvement in serum liver tests and also reduction in proinflammatory cytokines have been observed in nonalcoholic steatohepatitis related cirrhotics using VSL#3 [55].

On the other hand, in patients with primary sclerosing cholangitis, treatment with a probiotics cocktail containing four* Lactobacillus* and two* Bifidobacillus* strains did not improve clinical symptoms or liver function tests [56]. The authors attributed this lack of efficacy to the fact that all the PSC patients in the study were already in remission for their IBD, with limited scope for further improvement in IBD, and therefore PSC. As the majority of patients with PSC have concurrent inflammatory bowel disease (IBD) [57], toxic substances originating from the inflamed gut may also be the culprit for damaging the liver and biliary trees. It has already been established that probiotics are beneficial for IBD [58] and pouchitis [59]. It is therefore highly plausible that the same beneficial effect might extend to PSC. Nevertheless larger clinical studies are required before any conclusion can be drawn.

## 8. Nonalcoholic Fatty Liver Disease

Evidence in animal studies shows that intestinal bacterial overgrowth plays a significant role in the pathogenesis of nonalcoholic fatty liver disease (NAFLD) [60]. Furthermore, obese patients with bacterial overgrowth after jejunoileal bypass surgery experienced rapid worsening of their NAFLD [61], suggesting a causal link. Endotoxaemia worsens NAFLD by stimulating hepatic Kupffer cells to produce TNF-*α* which stimulates liver fibrosis [62].

Loguercio et al. demonstrated improvement in serum liver function tests and also reduction in proinflammatory cytokines in nonalcoholic steatohepatitis related cirrhotics using VSL#3 [55]. A Cochrane systemic review in 2007 concluded that, due to the lack of randomised controlled trials, the use of probiotics in NAFLD can neither be supported nor refuted [63]. Subsequent to that, Solga and Diehl examined four patients with NAFLD and assessed their liver fat after 4 months of VSL#3 therapy [64]. Disappointingly they found that all four patients experienced increase in liver fat as measured by proton magnetic resonance spectroscopy. More recently it has been shown that probiotics improve liver aminotransferases levels and reduce lipopolysaccharide levels in patients with NAFLD, although anthropometric parameters and cardiovascular risk factors remained unchanged after treatment [65, 66]. A larger study compared probiotics and fructooligosaccharides to life style changes in NAFLD with the probiotics arm significantly reducing TNF-*α*, CRP, serum AST levels, homeostasis model assessment of insulin resistance, serum endotoxin, steatosis, and the NASH activity index [67]. Long term use of probiotics may significantly reduce liver fat and serum aspartate aminotransferases [68]. Taking into account these newer studies, a recent meta-analysis concluded that probiotic therapies can reduce liver aminotransferases, total cholesterol, and TNF-*α* and improve insulin resistance in NAFLD patients [69]. However, these conclusions should be interpreted cautiously as the total number of patients involved is small, some patients are children, and the results are not based on histology, which is the gold standard for the diagnosis of NASH.

## 9. Alcoholic Liver Disease

Alcoholic steatohepatitis and severe alcoholic liver disease (ALD) occur in 30% of heavy drinkers [70], suggesting that other factors may also play a causative role. The pathogenesis of ALD is a dynamic and unknown process characterized by several interactions that involve immune system and metabolic intermediates of alcohol [71]. This includes the ethanol metabolism-associated oxidative stress, abnormal methionine metabolism, ethanol-mediated induction of leakage of gut endotoxins, and activation of Kupffer cells [72–74]. Chronic alcoholism is also associated with higher levels of Proteobacteria (Gram-negative bacteria which include several pathogenic species such as* Salmonella* and* Escherichia*) and lower abundances of Bacteroidetes [75]. The resultant endotoxaemia triggers the proinflammatory pathways causing alcoholic steatohepatitis.

Treatment with* Escherichia coli* Nissle probiotics has been shown to restore the intestinal microflora including* Lactobacilli* and* Bifidobacilli*, to reduce endotoxaemia, and to improve liver function [40]. This beneficial effect is confirmed in another larger study using a probiotic preparation containing* Bifidobacterium bifidum* and* Lactobacillus plantarum* [76]. Emerging data has also shown a beneficial effect of* Lactobacillus casei* Shirota in restoring neutrophil phagocytic capacity [77], a marker associated with increased risk of infection and mortality in ALD [78].

## 10. Portal Hypertension

Bacteria translocation plays a role in increasing portal pressure by contributing to the exacerbation of the hyperdynamic circulatory state and the increase in hepatic vascular resistance [79].

Utilising the measurement of hepatic venous pressure gradient (HVPG), relationships between portal hypertension and probiotics have been investigated. Use of adjunctive probiotics (VSL#3) increased the HVPG response rate (percentage of patients having a decrease from baseline of ≥20% or to ≤12 mm Hg) compared with propranolol alone and was similar to the response with adjunctive antibiotics. The mean fall in HVPG was greater with either adjunctive probiotics or adjunctive antibiotics than with propranolol alone [80]. A 6-week administration of VSL#3 resulted in reductions of the HVPG, as well as in the improvement of systemic haemodynamics including cardiac index and mean arterial pressure [81].

Data in this area is, however, conflicting. Two studies utilising VSL#3 did not reduce portal pressure in patients with compensated or decompensated cirrhosis. Furthermore, there were no significant changes in the stool microbiota evaluated by terminal restriction fragment length polymorphism, before and after therapy [79, 82].

## 11. Potential Risk

Although probiotics are generally well tolerated, even among cirrhotic patients [77], it is not without risk especially in patients with severe illness or in those who are immunocompromised. A study of patients with predicted severe acute pancreatitis given probiotic prophylaxis with a cocktail of six different bacteria was associated with an increased risk of mortality [83].

## 12. Conclusion

There is growing recognition that alteration of gut microbiota has a causative effect on the pathogenesis of numerous liver conditions including complications of liver cirrhosis. As a consequence, there is an increasing interest in the use of probiotics in preventing and treating these conditions. However, the role of probiotics in this context remains controversial. Emerging data are encouraging especially in the field of hepatic encephalopathy and NASH, although further studies are required before probiotics can be included in the respective treatment algorithms.
